# Combined aberrant expression of E-cadherin and S100A4, but not β-catenin is associated with disease-free survival and overall survival in colorectal cancer patients

**DOI:** 10.1186/1746-1596-8-99

**Published:** 2013-06-19

**Authors:** Sang-Jeon Lee, Song Yi Choi, Wun-Jae Kim, Meiying Ji, Taek-Gu Lee, Bo-Ra Son, Soon Man Yoon, Rohyun Sung, Eun Jeoung Lee, Sei Jin Youn, Seon Mee Park

**Affiliations:** 1 D1Department of Surgery, Chungbuk National University College of Medicine and Medical Research Institute, Cheongju, Chungbuk 361-763, Republic of Korea; 2 2Department of Pathology, Chungbuk National University College of Medicine and Medical Research Institute, Cheongju, Republic of Korea; 3 3Department of Urology, Chungbuk National University College of Medicine and Medical Research Institute, Cheongju, Republic of Korea; 4 4Department of Internal Medicine, Chungbuk National University College of Medicine and Medical Research Institute, Cheongju, Republic of Korea; 5 5Department of Laboratory Medicine, Chungbuk National University College of Medicine and Medical Research Institute, Cheongju, Republic of Korea

**Keywords:** Epithelial to mesenchymal transition, E-cadherin, β-catenin, S100A4, Tumor budding, Colorectal cancer

## Abstract

**Background/Aims:**

Epithelial-to-mesenchymal transition (EMT) in cancers is related to metastasis, recurrence, and poor prognosis. We evaluated whether EMT-related proteins can act as prognostic biomarkers in colorectal cancer (CRC) patients.

**Methods:**

We evaluated the expression of E-cadherin, β-catenin, and S100A4 by immunohistochemistry (IHC) in 333 CRC tissues from the tumor center and invasive margin. Tumor budding, cell grade, tumor stage, type of tumor growth, peritumoral lymphocyte infiltration (TLI), and perineural- or lymphovascular invasion were evaluated as pathological parameters. mRNA levels of E-cadherin, N-cadherin, β-catenin, and S100A4 from 68 specimens from the same set were analyzed by real time quantitative RT-PCR.

**Results:**

Loss of E-cadherin, nuclear β-catenin, and gain of S100A4 were higher in the invasive margin than in the tumor center. Loss of E-cadherin was associated with cell grade, macroscopic type, perineural invasion, and tumor budding, β-catenin with microsatellite instability and tumor site, and S100A4 with growth type, macroscopic type, AJCC stage, lymphovascular invasion, and perineural invasion. The aberrant expression of E-cadherin and S100A4 not β-catenin in the invasive margin was a significant and independent risk factor for disease-free and overall-survival by multivariate analysis, along with AJCC stage and perineural invasion. mRNA levels of β-catenin and S100A4 were correlated with the IHC findings at the tumor invasive margin. E-cadherin and N-cadherin showed a weak inverse correlation.

**Conclusions:**

The combination of loss of E-cadherin and gain of S100A4 in the tumor invasive margin can be used to stratify patients with the same AJCC stage into different survival groups.

**Virtual slides:**

The virtual slides for this article can be found here: http://www.diagnosticpathology.diagnomx.eu/vs/9398289629244673

## Background

The incidence of colorectal cancers (CRC) has been increasing in Korea since 1999. In 2009, CRC was the fourth most fatal cancer [1]. Although the 5-year survival rate of CRC overall has been reported to be as high as 71.3% [1], the survival rate in patients with recurrence is only 40% [2]. The recurrence rate of stage I - III CRC patients who received curative resection has been reported to be 27.3% [2]. In addition to American Joint Committee on Cancer (AJCC) stage, biomarkers to predict recurrence are needed to select those patients who should be treated more aggressively. The growth pattern of the invasive margin, tumor budding, tumor grade, perineural invasion, and lymphovascular invasion have been reported to predict a poor prognosis [3,4]. Tumor buds are thought to be responsible for the subsequent steps in invasion and metastasis [5]. They are considered the histological hallmark of the epithelial to mesenchymal transition (EMT) [6].

EMT is the process by which mature epithelial cells change in appearance and lose cell–cell contacts and epithelial protein expression while at the same time acquiring the phenotypic characteristics of mesenchymal cells [7]. Many different EMT-related proteins and transcriptional factors that promote tumor progression and local or distant metastasis have been reported. Immunohistochemical staining (IHC) of human tissues obtained from patients with CRC demonstrated that the loss or attenuation of epithelial marker expression and the gain of mesenchymal marker expression are closely related to tumor progression and poor prognosis.

The initial step in tumor invasion and metastasis is the break-up of adhesion junctions mediated by E-cadherin, resulting in extension of the tumor cells into the stroma and their attachment to the extracellular matrix. Loss of E-cadherin in CRC correlates with clinicopathologic features of aggressive CRC and predicts poor prognosis [8]. Dysfunction of the Wnt-signaling pathway plays an important role in colorectal carcinogenesis and Wnt signaling dysfunction leads to the nuclear accumulation of ß-catenin [9]. Nuclear translocation of β-catenin triggers an EMT and a proinvasive gene expression [10]. Nuclear β-catenin expression has been observed in advanced CRC, but the prognostic significance was not clarified; it was related to poor prognosis [11], no effect [9,12] or even favorable prognosis [13]. S100A4 is directly involved in the formation of metastasis from several different tumor types via increased cell motility and invasion [14]. In CRC, nuclear expression of this protein is related to advanced tumor stage [15] and poor metastasis-free and overall survival [16]. EMT-related proteins such as E-cadherin, β-catenin, and S100A4 are known to be related to carcinogenesis and tumor progression, but the relation of these protein expressions and whether these proteins can serve as prognostic biomarkers of CRC were not clarified.

The aim in this study was to evaluate whether EMT-related protein expression and clinicopathological features of CRC are useful prognostic predictors or not. We compared the patterns of EMT protein expression in the tumor center and invasive margin and determined if there were correlations between the IHC findings and mRNA expression levels of various EMT-related genes.

## Methods

### Patients and tissue samples

Paraffin-embedded tissues were obtained from the department of pathology and fresh frozen specimens were provided by the National Biobank of Korea, with the approval of the Ethics Committee of Chungbuk National University Hospital. Three hundred thirty-three CRC patients (male:female, 189:144), who underwent complete resection (R0) and were followed-up for more than 5 years were enrolled in this study. The patients did not receive any chemotherapy or radiation therapy before surgery. Among the enrolled patients, 68 fresh-frozen specimens were obtained for real time RT-PCR. At the time of surgery, tumor tissues and matched normal tissues were immediately sampled from the resected colorectal specimen by pathologists. The tissue was frozen in liquid nitrogen, and kept at −80°C.

### Histopathology

Each tumor was re-evaluated by analysis of the medical records and the tissue slide files by one pathologist. Tumor location (right side or left side), the degree of differentiation (well, moderately, and poorly), depth of tumor invasion, lymph node or distant metastasis, and microsatellite status (characterized in 166 cases) were assessed. The stages were defined according to the TNM staging system of AJCC. We also reviewed macroscopic type (polypoid, ulcerofungating, and ulceroinfiltrative), invasion to the lymphatics or vessels, and perineural invasion. Tumor growth was classified as expanding- or infiltrative-type and tumor budding was evaluated by cytokeratin staining. The number of tumor buds was counted in five regions of clusters of tumor cells comprising less than 5 cells at 200x magnification. We divided cases into those with low (median <10) or high budding (median ≥ 10) (Figure 1).

**Figure 1:** **Representative pathologic features of colorectal cancer.** Lymphovascular invasion (**A**), perineural invasion (**B**), lymphocyte infiltration (mild, moderate, and severe) (**C**), and type of tumor growth (expanding **D** and infiltrative **E**). High tumor budding at the invasive margin stained with hematoxylin and eosin (**F**) and cytokeratin expression (**G**).

### Tissue microarray (TMA) construction and immunohistochemistry (IHC)

After all slide reviews, 3-mm sized TMAs were constructed. Areas from the center and the invasive margin of the tumor with the lowest degree of differentiation but abundant in cells with high mitotic activity were chosen from the original blocks. These representative areas were marked by an experienced pathologist on hematoxylin and eosin (H&E)-stained slides from selected paraffin blocks. Serial 4-um sections were then cut from the TMA paraffin blocks. The sections were mounted on Capillary Gap plus Slides. Before IHC staining, all sections were deparaffinized and heated in citrate buffer (10 mM/L citric acid, pH 6.0) in a microwave oven. After inactivation by exposure to 3% H_2_O_2_ for 10 min, the sections were incubated with blocking serum at room temperature for 10 min. IHC staining was carried out using anti-E-cadherin (DakoCytomation, Glostrup, Denmark, 1:400), anti-cytokeratin (LeicaMicrosystems, Wetzlar, Germany, 1:300), anti-β-catenin (DakoCytomation, Glostrup, Denmark, 1:400) and anti-S100A4 (DakoCytomation, Glostrup, Denmark, 1:800) as primary antibodies. After incubation with secondary antibodies, the expression of these markers in cells was detected with diaminobenzidine (DAB; Sigma, St. Louis, MO, USA) by enhancement with a SABC kit (ZSGB-BIO, Beijing, China). Tissue sections stained without primary antibody served as a negative control. The slides were then counterstained with hematoxylin. The results were assessed by two pathologists who were blinded to the patients’ details. E-cadherin immunostaining was evaluated according to a method described previously [17]. E-cadherin staining was classified as grade 0 (preserved) when more than 90% of the CRC cells on a section showed strong membranous staining, or grade 1 (reduced or lost) when less than 90% of the CRC cells showed positive membranous staining. For β-catenin, the percentage of tumor cells with nuclear staining was evaluated and scored as grade 0 (0-30%) or grade 1 (30-100%). To evaluate S100A4 expression, staining intensity was recorded as 0 (no staining), 1 (weak staining), 2 (intermediate staining), or 3 (strong staining). The proportion of stained cells was expressed as a percentage. The staining score was obtained by multiplying the intensity and percentage of stained cells and classified as grade 0 (low expression) and grade 1 (high expression) (Figure 2).

**Figure 2:** **Immunohistochemical staining for E-cadherin, β-catenin, and S100A4 in colorectal cancers (×400).** E-cadherin, membranous staining at the center of the tumor (**A**, arrow) and loss or attenuation of expression at the invasive margin of tumor buds (**B**, arrow). β-catenin, membranous staining (**C**, arrow) and nuclear staining at the invasive margin of tumor buds (**D**, arrow). Negative (**E**, arrow) and positive (**F**, arrow) staining for S100A4.

### Real time quantitative RT-PCR of EMT related genes

Tumor and matched normal tissues were homogenized and total RNA was isolated using an RNeasy Mini kit (Qiagen, Tokyo, Japan) following the manufacturer’s instructions. All samples were treated with RNase-free DNase (Qiagen). RNA quality control and quantification were carried out on an Agilent 2100 Bioanalyzer using a RNA 6000 Pico LabChip (Agilent Technologies, Tokyo, Japan). First-strand complementary DNA was made from total RNA using the Prime Script RT-reagent kit (Amersham Biosciences Europe GmbH, Freiburg, Germany) according to the manufacturer’s instructions. To quantify the expression levels of E-cadherin, β-catenin, N-cadherin, and S100A4, real-time PCR amplification was performed with a Rotor Gene 6000 instrument (Corbett Research, Mortlake, Australia). Real-time PCR assays using SYBR Premix EX Taq (TAKARA BIO INC., Otsu, Japan) were carried out in micro-reaction tubes (Corbett Research, Mortlake, Australia). The PCR reaction was performed in a final volume of 10 μl, consisting of 5 μl of 2x SYBR premix EX Taq buffer, 0.5 μl of each 5’- and 3’- primer (10 pmol/μl), and 1 μl of sample cDNA. The product was 10-fold serially diluted from 100 pg/μl to 0.1 pg/μl. Dilution series of PCR products were used to establish standard curves for real-time PCR. Spectral data were captured by using Rotor-Gene Real-Time Analysis Software 6.0 Build 14 (Corbett Research, Mortlake, Australia). All samples were run in triplicate. Glyceraldehyde-3-phosphate dehydrogenase (GAPDH) was used as an endogenous RNA reference gene. Gene expression was normalized to the expression of GAPDH. Primers and product sizes for E-cadherin, N-cadherin, β-catenin, S100A4, and GAPDH are summarized in Table 1.

**Table 1:** Sequences of primers and product size used in real time RT-PCR

**Gene**	**Forward**	**Backward**	**size**
E-cadherin	AGTCACGCTGAATACAGTGG	CATTTTCTGGGCAGCTGATG	161
N-cadherin	CAGTGCAGTCTTATCGAAGG	GAAAGCTTCTCACGGCATAC	158
β-catenin	AATGGCAGTGCGTTTAGCTG	ATAGCACCTTCAGCACTCTG	233
S100A4	CACAAGTACTCGGGCAAAGA	TACACATCATGGCGATGCAG	211
GAPDH	TGAGAACGGGAAGCTTGTCA	GGAAGGCCATGCCAGTGA	258

### Statistical analysis

Differences were compared using Fisher’s exact test or Pearson’s test for qualitative variables and Student’s t-test or analysis of variance for continuous variables. Prognosis was determined by disease-free survival and overall survival. Prognostic factors were examined by univariate and multivariate analyses (Cox proportional hazards model). All statistical tests were two sided, and statistical significance was accepted at the P < 0.05 level. All analyses were performed using SPSS version 12.0 (SPSS Inc., Chicago, IL, USA).

## Results

### Clinicopathologic parameters related to EMT-related protein expression

Clinicopathologic characteristics of the patients showed in Table 2. The relation between clinicopathological parameters and aberrant expression of E-cadherin, β-catenin and S100A4 in the invasive margin was observed. Loss of E-cadherin was related with cell grade (p = 0.050), macroscopic type (p = 0.014), perineural invasion (p = 0.037) and high tumor budding (p = 0.010). Nuclear β-catenin expression was higher in microsatellite stable (MSS) than microsatellite instable (MSI) tumors (p = 0.004) and left CRCs than in right CRCs (p = 0.037). S100A4 expression was increased in infiltrative growth (p = 0.017), macroscopic type (p = 0.024), T-stage (p = 0.010), nodal stage (p = 0.002), AJCC stage (p = 0.001), ratio of metastatic lymph nodes (p = 0.019), lymphovascular invasion (p = 0.034), and perineural invasion (p = 0.050). It was also related with TLI (p = 0.001) (Table 3).

**Table 2:** Clinical and pathological characteristics of 333 patients with colorectal cancers

**Characteristics**	**N (%)**
Age (years), Mean ± SD (range)	63.6 ± 11.1 (25-86)
Gender	
Male	189 (56.8)
Female	144 (43.2)
Tumor Grade	
Well	77 (23.1)
Moderately	236 (70.9)
Poorly	11 (3.3)
Undetermined	9 (2.7)
Depth of Invasion	
T1	13 (3.9)
T2	43 (12.9)
T3	210 (63.1)
T4	67 (20.1)
Nodal Stages	
N0	195 (58.6)
N1(a, b)	86 (25.8)
N2(a, b)	52 (15.6)
AJCC stage	
I	44 (13.2)
II	143 (42.9)
III	119 (35.7)
IV	27 (8.1)
Lymphovascular Invasion	
Negative	240 (72.1)
Positive	93 (27.9)
Perineural invasion	
Negative	306 (91.9)
Positive	27 (8.1)
Lymphocyte infiltration	
Mild	112 (33.6)
Moderate	170 (51.1)
Severe	45 (13.5)
Type of Tumor Growth	
Expanding	118 (36.3)
Infiltrative	207 (62.2)
Undetermined	8 (2.4)
Tumor budding	
Yes	44 (13.2)
No	289 (86.8)

**Table 3:** Relation between clinico-pathological parameters and immunohistochemistry of E-cadherin, β-cadherin, and S100A4 at invasive margin in colorectal cancers (n = 305)

**Parameters**	**E-cadherin**		**P**	**β-cadherin**		**P**	**S100A4**		**P**
	**Strong (n = 208)**	**Weak or Loss (n = 97)**		**Nuclear, Low (n = 267)**	**Nuclear, High (n = 38)**		**Low (n = 267)**	**High (n = 267)**	
Preoperative CEA (ng/ml)	7.0 ± 22.5	6.5 ± 12.4	0.811	6.5 ± 19.8	8.4 ± 18.3	0.573	5.3 ± 13.1	12.5 ± 35.7	0.014
MSI status (n = 166)			0.167			0.004			0.386
MSI-H (n = 8)	3(37.2)	5(62.5)		8(100.0)	0(0.0)		7(87.5)	1(12.5)	
MSI-L (n = 6)	3(50.0)	3(50.0)		4(66.7)	2(33.3)		5(83.3)	1(16.7)	
MSS (n = 135)	91(67.4)	44(32.6)		107(81.1)	25(18.9)		107(80.5)	26(19.5)	
Tumor Location			0.455			0.037			0.704
Right (n = 66)	48(72.7)	18(27.3)		*6.5 ± 18.7			60(87.0)	9(13.0)	
Left (n = 236)	158(66.9)	78(33.1)		*12.2 ± 22.7			194(84.0)	37(16.0)	
Tumor Budding			0.011			0.799			0.480
Low (<10) (n = 263)	188(70.9)	77(29.1)		230(87.1)	34(12.9)		224(85.2)	39(14.8)	
High (≥ 10) (n = 40)	20(50.0)	20(50.0)		37(90.2)	4(9.8)		32(80.0)	8(20.0)	
Macroscopic Tumor Type			0.616			0.909			0.038
Polypoid (n = 21)	17(77.3)	5(22.7)		18(85.7)	3(14.3)		21(100.0)	0(0.0)	
Ulcerofungating (n = 160)	109(66.9)	54(33.1)		143(88.3)	19(11.7)		138(86.3)	22(13.8)	
Ulceroinfiltrative (n = 122)	82(68.3)	38(31.7		106(86.9)	16(13.1)		97(79.5)	25(20.5)	
Tumor Grade			0.735			0.817			0.577
Well (n = 73)	53(72.6)	20(27.4)		64(86.5)	10(13.5)		60(82.2)	13(17.8)	
Moderate or Poor (n = 227)	151(66.5)	73(34.0)		196(87.5)	28(12.5)		191(85.3)	33(14.7)	
Ratio of Metastatic Lymph Node	0.11 ± 0.19	0.13 ± 0.21	0.567	0.12 ± 0.20	0.09 ± 0.19	0.317	0.11 ± 0.19	0.18 ± 0.23	0.019
Nodal Stages			0.567			0.288			0.002
N0 (n = 178)	128(70.3)	54(29.7)		155(85.2)	27(14.8)		161(90.4)	17(9.6)	
N1 (n = 77)	49(63.6)	28(36.4)		69(92.0)	6(8.0)		57(74.0)	20(26.0)	
N2 (n = 48)	31(67.4)	15(32.6)		43(89.6)	5(10.4)		38(79.2)	10(20.8)	
Depth of Invasion			0.513			1.000			0.010
T1, T2 (n = 50)	38(73.1)	14(26.9)		44(88.0)	6(12.0)		48(96.0)	2(4.0)	
T3, T4 (n = 253)	170(67.2)	83(32.8)		223(87.5)	32(12.5)		208(82.2)	45(17.8)	
AJCC stage			0.272			0.669			0.001
I (n = 39)	27(67.5)	13(32.5)		35(87.5)	5(12.5)		37(94.9)	2(5.1)	
II (n = 133)	96(71.1)	39(28.9)		114(85.1)	20(14.9)		119(89.5)	14(10.5)	
III (n = 110)	74(68.5)	34(31.5)		97(89.8)	11(10.2)		81(73.6)	29(26.4)	
IV (n = 21)	11(50.0)	11(50.0)		21(91.3)	2(8.7)		19(90.5)	2(9.5)	
Lymphovascular Invasion			0.891			0.341			0.050
Negative	150(68.5)	69(31.5)		195(88.6)	25(11.4)		189(87.1)	28(12.9)	
Positive	57(67.1)	28(32.9)		72(84.7)	13(15.3)		66(77.6)	19(22.4)	
Neural Invasion			0.037			0.507			0.050
Negative	196(69.8)	85(30.2)		248(87.9)	34(12.1)		240(85.7)	40(14.3)	
Positive	11(47.8)	12(52.2)		19(82.6)	4(17.4)		15(68.2)	7(31.8)	
Lymphocyte infiltration			0.325			0.821			< 0.0001
Mild	70(72.9)	26(27.1)		88(88.9)	11(11.1)		70(71.4)	28(28.6)	
Moderate	108(67.1)	53(32.9)		138(86.3)	22(13.8)		144(89.4)	17(10.6)	
Severe	26(60.5)	17(39.5)		36(87.8)	5(12.2)		38(95.0)	2(5.0)	
Type of Tumor Growth			0.159			1.000			0.044
Expanding	79(73.1)	29(26.9)		93(87.7)	13(12.3)		96(90.6)	10(9.4)	
Infiltrative	125(65.1)	67(34.9)		168(87.0)	25(13.0)		156(81.3)	36(18.8)	

Lymph Node Ratio, number of metastatic lymph nodes / number of harvested lymph nodes; *CEA* carcinoembryonic antigen serum level, *, percentage of β-catenin nuclear expression at invasive margin.

### Relation of E-cadherin,β-catenin and S100A4 expression

The aberrant expression of EMT-related proteins was higher in the invasive margin than in the tumor center; loss of E-cadherin, 17.9% versus 31.8% (p < 0.0001), nuclear expression of β-catenin, 10.6% versus 12.5% (p < 0.0001), and gain of S100A4, 10.2% versus 15.5% (p < 0.0001), respectively. Aberrant expression of each protein was related to the others: S100A4 versus E-cadherin (r = 0.312, p = 0.050), S100A4 versus β-catenin (r = 0.166, p = 0.004) and E-cadherin versus β-catenin (r = 0.152, p = 0.009).

### Prognostic factors of disease-free survival and overall survival

Disease-free survival was associated with AJCC stage (p < 0.0001, Figure 3A), tumor budding (p = 0.007, Figure 3B), tumor growth type (p = 0.003, Figure 3C), and perineural invasion (p = 0.004, Figure 3D). Aberrant expression of the E-cadherin (p = 0.007, Figure 3E), S100A4 (p = 0.004, Figure 3F), and combination of both proteins in the invasive margin were related to disease free survival (p = 0.005, Figure 3G), whereas β-catenin was inversely related (p = 0.032, Figure 3H). Multivariate Cox analysis showed that combination of E-cadherin and S100A4 expressions in the invasive margin and the AJCC stage are independent risk factor for disease-free survival (Table 4). Overall survival was associated with AJCC stage (p < 0.0001, Figure 4A), tumor budding (p = 0.01, Figure 4B), tumor growth type (p = 0.01, Figure 4C), perineural invasion (p = 0.02, Figure 4D), and TLI (p = 0.005, Figure 4E). Aberrant expression of E-cadherin (p = 0.002, Figure 4F), S100A4 (p = 0.003, Figure 4G), and combination of both proteins in the invasive margin were associated with overall survival time (p = 0.0002, Figure 4H), whereas β-catenin was not. Cox regression analysis showed that the combination of E-cadherin and S100A4 in the invasive margin, the AJCC stage and perineural invasion were independent risk factors of overall survival time (Table 5).

**Figure 3:** **Analysis of disease free survival time according to histopathologic parameters and EMT related protein expression.** AJCC stage (**A**), tumor budding (**B**), type of tumor growth (**C**), Perineural invasion (**D**), E-cadherin expression (**E**), S100A4 expression (**F**), combination of E-cadherin and S100A4 (**G**), and β-catenin expression (**H**).

**Table 4:** Cox regression analysis for disease free survival time in colorectal cancers

**Parameters**	**P value**	**Hazard Ratio**	**95% CI**
*EMT, invasive front	0.026	1.60	1.01-2.43
Lymphovascular invasion	0.625	1.15	0.90-4.28
Perineural invasion	0.092	1.96	0.90-4.28
Lymphocyte infiltration	0.987	1.00	0.66-1.52
Tumor growth type	0.306	1.43	0.72-2.85
Tumor budding (≥10/x200HPF)	0.168	1.61	0.82-3.15
AJCC stage	0.000	3.03	2.03-4.52

*EMT included the expressions of E-cadherin and S100A4.

**Figure 4:** **Analysis of overall survival time according to histopathologic parameters and EMT related protein expression.** AJCC stage (**A**), tumor budding (**B**), type of tumor growth (**C**), Perineural invasion (**D**), Peritumoral lymphocytic infiltration (TLI) (**E**), E-cadherin expression (**F**), S100A4 expression (**G**), and combination of E-cadherin and S100A4 (**H**).

**Table 5:** Cox multivariate analysis for overall survival time in colorectal cancers

**Parameters**	**P value**	**Hazard Ratio**	**95% CI**
*EMT, invasive front	0.036	1.54	1.03-2.31
Lymphovascular invasion	0.963	1.01	0.58-1.78
Perineural invasion	0.010	2.58	1.25-5.34
Lymphocyte infiltration	0.696	0.92	0.60-1.41
Tumor growth type	0.119	1.73	0.87-3.44
Tumor budding (≥10/x200HPF)	0.778	0.90	0.60-1.41
AJCC stage	0.001	1.84	1.26-2.68

*EMT included the expressions of E-cadherin and S100A4.

### Association between mRNA expression and IHC findings

Transcript levels of β-catenin and S100A4 were correlated with IHC findings at the tumor invasive margin; β-catenin (r = 0.369, p = 0.003) and S100A4 (r = 0.504, p < 0.0001). However, there was no relation between the RT-PCR data and the IHC findings for E-cadherin. E-cadherin and N-cadherin showed a weak inverse relation without statistical significance (r = -0.169, p = 0.084). mRNA levels of N-cadherin were higher in recurrent or mortality cases (p = 0.040 and p = 0.042, respectively).

## Discussion

In this study, we demonstrated that the combination of the loss of E-cadherin and gain of S100A4 in the invasive margin of CRC is an independent prognostic factor of a poorer outcome, along with AJCC stage and perineural invasion. Nuclear expression of β-catenin was not related to patient survival.

When tumor cells start to invade and metastasize, adhesion molecules undergo alterations. Down-regulation of E-cadherin in CRC is associated with malignant features. Loss of E-cadherin has been shown to be associated with tumor budding [18] and lymph node metastasis in CRC [19] and to predict disease recurrence and long-term survival in CRC [8,20,21]. In this study, loss of E-cadherin at the invasive margin of CRCs was associated with high tumor budding, perineural invasion, and a poor prognosis.

S100A4 is localized in the nucleus, cytoplasm, and extracellular space and has a wide range of biological functions ranging from regulation of angiogenesis to cell survival, motility, and invasion [14]. We found that S100A4 expression in the invasive margin was increased in infiltrative tumors, those with a lymph node metastasis, advanced AJCC stage, or lymphovascular- and perineural invasion, which are all parameters representing tumor aggressiveness. We demonstrated that high expression of S100A4 is associated with recurrence and mortality. These results were consistent to the previous studies [15,22,23], in which S100A4 is related to a poor prognosis. One study reported that S100A4 is overexpressed in cell populations enriched for stem-like cells, which is associated with Wnt/APC/β-catenin signaling pathway and S100A4 worked as β-catenin/TCF target gene [24]. Inconsistently other results, S100A4 was also related to lymphocyte infiltration, which protects tumor progression and destroys tumor budding. These findings were resulted from that S100A4 expressing fibroblasts, monocytes, macrophages, T lymphocytes, neutrophilic granulocytes, or endothelial cells may be misinterpreted as S100A4 expressing cancer cells [14].

β-catenin plays to maintain cell-to-cell adhesion along with E-cadherin. However, β-catenin also acts as a transcription factor in the Wnt signal transduction pathway and Wnt signaling dysfunction leads to the nuclear accumulation of ß-catenin [9]. Several studies have reported that nuclear ß-catenin expression in the invasive margin is associated with high tumor budding and poor prognosis [11], whereas other studies did not find such a relationship [9,12,20]. In addition, recent study showed that aberrant β-catenin expression was related to favorable prognosis [13]. We did not find any association between β-catenin expression and tumor budding or overall survival in our patient cohort. These inconsistencies may result from different CRC subtypes, the existence of more than one type of CRC in a study [25], or different evaluation methods [3]. We showed that β-catenin nuclear expression was increased in MSS tumors compared to MSI tumors and that it was higher in left CRCs than right CRCs. These results are consistent with those of a previous study [26], which reported that MSI-high, *CpG island methylator phenotype (CIMP)*-high, and BRAF mutations, which are characteristics of right CRCs, showed an inverse association with cytoplasmic and nuclear β-catenin expression. MSS and MSI colorectal cancers are increasingly being recognized as distinct entities with significantly different pathological characteristics, behaviors, and prognoses [27]. MSI is associated with significantly lower levels of nuclear ß-catenin and impaired EMT than MSS [27]. In agreement with these reports, we found that 44.4% of MSI-H cases versus 72.4% of MSS or MSI-L cases were tumor budding positive.

Aberrant expression of E-cadherin, β-catenin, and S100A4 showed parallel patterns each other. These results suggested that overexpression of S100A4 inhibits E-cadherin expression and β-catenin plays a role in driving S100A4-dependent EMT induction [14]. Although individual change of E-cadherin and S100A4 was related to patients’ prognosis in univariate survival analysis, multivariate Cox analysis revealed that the combination of E-cadherin loss and S100A4 overexpression was the only prognostic factor in addition to AJCC stage, which is still the most important prognostic factor in CRC. These results highlight the fact that multi-marker phenotypes rather than single protein are needed in IHC biomarker investigations [3].

Because the tumor biology of the invasive margin is different than that of the tumor center, the patterns of EMT protein expression are expected to be different at the two sites. In this study, EMT-related changes in the expression of E-cadherin, β-catenin and S100A4 were more severe in the invasive margin than in the tumor center and EMT changes in the invasive margin, but not the tumor center, had prognostic significance.

Tumor budding is a putative hallmark of CRC cell invasion and has previously been shown to be associated with various clinicopathological parameters, including lymph node metastasis, vascular and lymphatic invasion, distant metastasis, local recurrence, and poor outcomes [28]. In this study, high tumor budding was associated with the ratio of metastatic lymph nodes, type of tumor growth, and perineural invasion (data not shown). It has also been classified as an additional prognostic factor. However, our results suggest that the combination of E-cadherin and S100A4 expression at the invasive margin of CRC is superior to tumor budding for predicting prognosis.

The mRNA levels of E-cadherin, β-catenin, and S100A4 were not found to be associated with histopathological parameters or prognosis in this study. For β-catenin and S100A4, mRNA levels reflected that of the encoded protein, but this was not the case for E-cadherin. However, the switch in expression from E-cadherin to N-cadherin and the higher expression of N-cadherin in patients with a poor prognosis were demonstrated in this study. Recent study also showed that N-cadherin was highly expressed in type II papillary renal cell carcinomas than type I cancers and type II cancers were related to poor prognosis [29].

In conclusion, our results suggest that aberrant expression of E-cadherin and S100A4 in the invasive margin was well related with clinicopathological parameters and IHC of both proteins is useful marker to predict prognosis in CRC.

## Abbreviations

AJCC: American Joint Committee on Cancer; CRC: Colorectal cancer; EMT: Epithelial-to-mesenchymal transition; GAPDH: Glyceraldehyde-3-phosphate dehydrogenase; IHC: Immunohistochemistry; H&E: Hematoxylin and eosin; MSI: Microsatellite instability; MSS: Microsatellite stable; TLI: Peritumoral lymphocyte infiltration; TMA: Tissue microarray

## Competing interests

The authors declare that they have no competing interests.

## Authors’ contributions

S-JL contstructed the manuscript. SYC and RS carried out pathologic study. W-JK checked mRNA levels. MJ constructed tissue microarray. T-GL, B-RS, SMY, and SJY were responsible for clinical data. SMP designed and constructed manuscript. All authors read and approved the final manuscript.
